# A Data-Driven Medical Decision Framework for Associating Adverse Drug Events with Drug-Drug Interaction Mechanisms

This article has been retracted.

**DOI:** 10.1155/2022/9132477

**Published:** 2022-03-03

**Authors:** Adeeb Noor

**Affiliations:** Information Technology Department, Faculty of Computing and Information Technology, King Abdulaziz University, Jeddah 21589, Saudi Arabia

## Abstract

Adverse drug events (ADEs) occur when multiple drugs interact within an individual, thus causing effects that were not initially predicted. Such toxic interactions lead to morbidity and mortality. Contemporary research surrounding ADEs has tended to focus on the detection of potential ADEs without great concern for elucidating the associations of drug-drug interaction (DDI) mechanisms that can predict potential adverse drug reactions (ADRs). Such associations are of great practical importance for everyday pharmacovigilance efforts. This study presents a data-driven framework for conducting knowledge-driven data analysis that combines a semantic inference system and enrichment analysis in order to identify potential ADE mechanisms. The framework was used to rank mechanisms according to their relevance for DDIs and also to categorize ADEs based on the number of DDI mechanism associations identified through enrichment analysis. Its validity is demonstrated through using both commercial and publicly available DDI resources. The results of this study solidly prove the framework's effectiveness and highlight potential for future research by way of incorporating additional and broader data to deepen and expand its capabilities.

## 1. Introduction

One type of medical error is adverse drug events (ADEs), the occurrence of which is recognized as among the greatest concerns in cases of drug-drug interaction (DDI). ADEs occur when multiple drugs interact within an individual to cause unanticipated toxic effects, which lead to morbidity and mortality. As reported in multiple studies [1–3], ADEs cause considerable illness and death; they kill over 770,000 patients in U.S. hospitals each year, with an estimated annual cost of $5.6 million per hospital [4, 5]. While additional ADEs may be prevented by contraindicating drug pairs that have been observed to generate toxic interactions in a clinical setting, new approaches are required to predict and prevent never-before-seen ADEs.

Fundamentally, multiple avenues can be pursued when endeavoring to study and understand ADEs. Traditional ADE research efforts are bench-science-based, i.e., conducted either in vivo (in living organisms) or in vitro (outside living organisms). While such studies are important, their scope is narrow; effective avoidance of ADEs requires the collection and integration of comprehensive knowledge regarding diseases, targets, drugs, drug effects, and underlying interaction mechanisms. Accordingly, the field of pharmacovigilance (PhV) was introduced by the World Health Organization to monitor, collect, and synthesize research information from multiple resources, the better to prevent short-term and long-term side effects resulting from ADEs [6]. PhV implementations have shown promising results in studying and predicting ADEs before their occurrence, for example, through data extraction, collection, and creation [7–10]. Other applications have focused on predicting ADEs using computational methods such as text mining [11], machine learning [12], deep learning [13], and network models [14]. Such methods often employ inputs that are clinically based, such as electronic patient records [15], clinical notes [16], disease characteristics [17], or drug features [18]; other nonclinical inputs consist of personal messages [19], social media posts [20], and advice from human experts [21]. Overall, these studies have concentrated more strongly on identifying new potential ADEs rather than providing support for determination of the mechanisms of drug interaction.

Examining ADEs within the context of their defining mechanisms, which stem from DDIs, is one of the most potent methods for advancing our understanding. In that regard, two main approaches have been undertaken. The first is a drug-based approach, in which the features or relations of drugs related to ADEs are studied and analyzed in order to uncover ADE mechanisms; for example, studies have examined drugs and their molecular targets [22], drug properties such as chemical substructure [23], and drug-target relationships [24]. The second approach centers on ADEs and is geared toward studying and understanding disease/phenotype profiles and gene-pathway interactions [25]. Both approaches have shown promising outcomes in terms of advancing prediction of ADEs prior to their occurrence, but they also share two important limitations, focusing on either drug-ADE or phenotype-ADE relations and considering only pharmacokinetic or pharmacodynamic mechanisms. In addition, discovery of ADEs involves a careful combination of analyses, integrating data from diverse sources with knowledge of underlying interaction mechanisms [26]. Combining established approaches with knowledge of the many possible DDI mechanisms is essential to informing strategies for ADE prevention [27]. The ultimate aim of this work is to illustrate the potential for advancement of ADE research by leveraging the data and knowledge regarding DDI mechanisms contained within multiple biomedical repositories to fill gaps and potentially predict ADEs.

Here, we present a data-driven medical decision framework developed to perform knowledge-driven data analysis to associate mechanisms of ADEs together with DDIs. Specifically, our framework relies on structured knowledge and ontology-based annotations in conjunction with a semantic inference system to associate ADEs with ten correlated DDI mechanisms, allowing for categorization of ADEs through enrichment analysis. We conducted two demonstrative experiments with this framework, first, ranking mechanisms according to their relevance for DDIs and, second, generating ten corresponding ADE datasets and using them in enrichment analysis. We also demonstrate our framework using both commercial and publicly available DDI resources and show how it can aid clinicians in identifying patients at risk of ADEs stemming from DDIs, including ADEs that have yet to be fully characterized.

## 2. Materials and Methods

The framework is designed around utilizing experimental data from the Human Phenotype Ontology (HPO) [28] in conjunction with the drug-drug interaction discovery and demystification (D3) inference framework by Noor et al. [29]. It ranks the predictive significance of DDI mechanisms and explores the associations of ADEs with potentially correlated DDI mechanisms, allowing categorization of ADEs.  Table 1 shows the mechanisms of interaction covered by the D3 framework. Two experiments are presented here, each employing the system in a different capacity to showcase some of the inferences it could be used to draw and each designed to yield outcomes of potential direct benefit to clinicians. These are not intended to exhibit the full capacity of what is possible with this system, leaving room for future expansion beyond the framework presented herein.

### 2.1. Experiment (1): Rank the Predictive Significance of DDI Mechanisms

The first experiment was designed to first construct annotations that associate interacting drug pairs with DDI mechanisms and then apply an extra trees' classifier to rank those mechanisms (features) according to predictive significance. A total of 146 drug pairs (73 interacting and 73 noninteracting) were retrieved manually from Micromedex, a well-known commercial DDI repository, without consideration for potentially applicable DDI mechanisms. A pharmacist was then asked to review all 146 drug pairs. Each drug was then manually mapped to its respective concept unique identifier (CUI) in Unified Medical Language System (UMLS) [37] as required by the D3 inference framework, which was used to confirm and annotate the interactivity or noninteractivity of each pair. Next, a feature matrix was constructed in which rows contained drug pairs and columns contained the applicability of distinct DDI mechanisms. Finally, the extra trees' classifier was applied to the matrix, with 70% of the set used for training and 30% for testing.

An extra trees' classifier is akin to a random forest, but more extreme. In this classifier, several randomized decision trees are fitted to multiple independent subsamples, the results of which are averaged to limit overfitting and increase prediction accuracy. As with a random forest classifier, extra trees select a random sample from among the candidate features. Rather than identifying thresholds that provide greatest discrimination, however, extra trees randomize the threshold for each feature and use the best-performing threshold to define the splitting rule. This approach typically enables the model's variance to be reduced somewhat further, though with the tradeoff of slightly increasing bias.

In the classifier, the relative rank (i.e., depth) of any given decision node (i.e., feature) represents its relative importance in predicting the target variable; that is, features positioned higher in the tree contribute to prediction decisions for a greater portion of the input dataset. Accordingly, a feature's relative importance can also be estimated in terms of the expected fraction of samples for which it contributes to prediction decisions (i.e., the expected activity rate). Generating multiple randomized trees and averaging a feature's expected activity rates across them reduces the variance of its estimated importance, which is useful in feature selection.  Figure 1 shows the workflow for ranking features (mechanisms) using the extra trees classifier.

### 2.2. Experiment (2): Categorize ADEs by the Count of DDI Mechanism Associations

In this second scenario, the semantic inferences from experiment (1) and an ontology were used to associate DDI mechanisms with ADEs and categorize them via enrichment analysis. Specifically, enrichment analysis was carried out over the HPO, where each term explains a phenotype deviation, and ADEs in the ontology were examined for enrichments of the ten DDI mechanisms from the D3 inference framework. This experiment was comprised of four essential steps (Figure 2).

1. First, TWOSIDES [9], a repository of FDA-recognized spontaneous ADEs containing 63,473 unique interacting drug pairs (645 drugs and 1318 ADEs), was chosen as a dataset due to being freely available to the public and providing a sufficient number of DDI-ADE associations with corresponding likelihood values (*p* values).
2. Second, TWOSIDES was annotated with DDI mechanism information using the D3 inference framework; specifically, all drugs listed in TWOSIDES were mapped to UMLS CUIs; then, each drug pair was fed through the D3 framework. The recall rate for the overall inferential coverage of TWOSIDES was computed, with the result being above 79% (49,915 inferred interactions out of 62,886 verified interactions). This value is critical for computing the recall rates associated with individual DDI mechanisms.
3. Third, enrichment analysis was used to rank the predictive significance of the associations between DDI mechanisms and ontological annotations in the HPO. The ADEs in TWOSIDES (represented by UMLS identifiers) were mapped to HPO terms using a Java OWL script. ADE test sets were then constructed for each of the ten DDI mechanisms, with each having a Boolean outcome based on detection of a DDI within the set by the D3 framework. Subsequently, the ontology analysis tools FUNC [38] (used to find associations specifically with Gene Ontology terms) and OntoFunc [39] (used for different ontologies) were leveraged to carry out enrichment analysis and rank associations between the ten DDI mechanisms and the HPO annotations for ADEs. This yielded ten annotated sets, each consisting of three columns: DDI, phenotype (ADE) from the HPO, and the Boolean result of the inference drawn by the D3 framework.
4. Finally, a hypergeometric test was performed on the ten annotated records to assess the probability of “drawing” the observed number of differentially expressed ADEs for each mechanism.

We also employed the Wilcoxon signed-rank test to identify the quality of the ten mechanisms in terms of distinguishing between positive and negative DDIs in TWOSIDES. For each DDI pair found to be associated with multiple ADEs, we chose the association having the smallest nonzero *p* value. The Wilcoxon test was run in *R* and a W value of 3843500 and a median difference between positive and negative DDIs of 0.04692435 (95% confidence interval 0.0377504–0.0541043 and *p* value < 2.2e-16) were returned.

## 3. Results and Discussion

### 3.1. Ranking Mechanisms according to Their Relevance for DDIs

The first experiment considered a total of 146 drug pairs (73 interacting and 73 noninteracting; 70% used for training and 30% for testing) and ranked the predictive significance of DDI mechanisms.  Table 2 summarizes the results of this experiment.

In this ranking of predictive significance, the framework demonstrated good capability overall: average precision 0.855, average recall 0.866, and average F1 score 0.855. The F1 scores obtained for each DDI mechanism were metabolic inhibition, 0.281019, metabolic induction, 0.242089, protein binding, 0.168295, multipathway, 0.109771, side-effect similarity, 0.091208, indication similarity, 0.047006, transporter inhibition, 0.034505, transporter induction, 0.022949, additive pharmacodynamic, 0.003157, and competitive pharmacological, 0.000000.

### 3.2. Enrichment Analysis over HPO terms to Identify Which ADEs Are Associated with Each DDI Mechanism

Before running the enrichment analysis, we examined the individual recall rates of the ten mechanisms for ADEs in TWOSIDES. Mutual exclusivity of the asserted DDIs was not incorporated, that is, in the event of multiple mechanistic explanations for a given DDI, that DDI was counted towards all relevant inferences. The F1 scores per mechanism were side-effect similarity, 0.76, metabolic inhibition, 0.29, protein binding, 0.21, transporter inhibition, 0.13, metabolic induction, 0.11, multipathway, 0.08, indication similarity, 0.06, transporter induction, 0.03, competitive pharmacological, 0.02, and additive pharmacodynamic, 0.01.

We next performed enrichment analysis over HPO terms to identify which ADEs among the ontology associate with each mechanism. This analysis yielded several examples of significant ADEs involving medications that share one or more of the listed mechanisms; for example, thrombocytopenia (*p* = 6.13E-06) was identified as a common ADE that can be a direct risk for medications sharing the same indication (cf. Tirofiban and abciximab, or quinine and quinidine) [40–42].

To further characterize the associations of DDI mechanisms with ADEs, we categorized ADEs based on the number of associated mechanisms. From each DDI mechanism, we picked the top ten associations having the lowest *p* values, which yielded 55 examples of potentially significant ADEs. We then tabulated the number of DDI mechanisms associated with each ADE (Table 3). The most prominent was “abnormality of inflammatory response,” which was associated with six DDI mechanisms; another eleven ADEs were each associated with five mechanisms. The complete per-mechanism results are reported in Supplementary 1.

In addition to potentially predicting ADEs that could result in noxious ADRs, this approach opens avenues for providing some indication of their frequency, which could aid clinicians in identifying at-risk patients. However, an important limitation to consider is data availability. When designing a data-driven system, the quantity of training data can potentially be limited by available financial and material resources, as well as the scope of the design. In regard to commercial repositories of DDI mechanisms, readily available data can be quite constrained by factors including limited sharing, limited research, and private control of information. Such limitations are a driving force behind the construction of computational systems; this study was impelled by the apparent lack of an automated resource for evaluating the effectiveness of such systems from a clinical standpoint. Considering that one of the primary goals in designing this framework was to raise the standard of research by only associating DDI mechanisms with clinically proven ADEs, it was necessary to base the training data on highly reliable information from clinical sources and medical practice. This led to the use and reuse of established knowledge repositories and consequently leveraging collective information from multiple resources. Notably, the knowledge sources employed here were by no means comprehensive given the many other high-quality sources available. Rather than constituting a limit of this framework, however, the existence of such additional sources offers opportunities for its future expansion. For one, the depth, precision, and recall can be improved by way of additional training data. Similarly, incorporating additional types of information that lead to expanded annotations can extend the breadth of inferences and classifications. This framework should not be construed as an end goal; indeed, it should ideally lead to its own obsolescence if the inferences used to draw prove of significant aid in expanding the known associations of DDI mechanisms with ADRs.

## 4. Conclusions

This study developed a data-driven medical decision framework for identifying potential ADE mechanisms and anticipating potential ADRs in a knowledge-driven manner. The framework combines a semantic inference system and enrichment analysis and is distinct from extant efforts in approaching the problem from the perspectives of drugs and diseases. Here, the framework was employed first to rank DDI mechanisms and second to relate ADEs to DDI mechanisms based on data from commercial and publicly available resources. Its performance was further evaluated on patient health records from TWOSIDES, in which the framework demonstrated good performance at grouping ADEs with known mechanisms. Overall, the results of these tasks support this framework as being a potentially useful tool for clinicians and researchers alike.

## Figures and Tables

**Figure 1:** Overall steps in the process of ranking DDI mechanisms.

**Figure 2:** Workflow for applying enrichment analysis over ADEs with semantic inference to identify mechanisms.

**Table 1:** Proposed mechanisms of drug-drug interaction according to the D3 framework [29].

#	Mechanism	Definition
1	Protein binding [30]	Displacement reactions between two drugs
2	Metabolic induction [31]	Induction is caused by one of two drugs
3	Metabolic inhibition [31]	Inhibition is caused by one of two drugs
4	Transporter induction [32]	Induction is caused by one of two drugs
5	Transporter inhibition [32]	Inhibition is caused by one of two drugs
6	Multiple pathways [33]	Both drugs share enzymes and transporters
7	Competitive pharmacological [34]	Both drugs share a target
8	Additive pharmacodynamic [35]	Both drugs share mechanisms of action
9	Indication similarity [36]	Both drugs treat the same disease
10	Side-effect similarity [31]	Both drugs share side effects

**Table 2:** Performance metrics obtained when using the extra trees' classifier on 146 commercially recognized DDI pairs.

	Precision	Recall	F1 score
Interacting drug pairs (73)	0.79	0.88	0.83
Noninteracting drug pairs (73)	0.92	0.85	0.88

**Table 3:** Selected potentially significant ADEs and corresponding counts of associated DDI mechanisms.

No. of associations	ADEs (HPO)
6 mechanisms	Abnormal inflammatory response
5 mechanisms	Neurological speech impairment
	Dysphonia
	Abnormality of body weight
	Pancreatitis
	Abnormality of leukocytes
	Abnormality of bone marrow cell morphology
	Abnormality of erythrocytes
	Abnormality of cells of the erythroid lineage
	Pancytopenia
	Abnormality of multiple cell lineages in the bone marrow
	Thrombocytopenia
4 mechanisms	Abnormality of higher mental function
	Growth abnormality
	Decreased body weight
3 mechanisms	Abnormal emotion/affect behaviour
	Restlessness
	Thrombophlebitis
	Venous thrombosis
	Diabetes mellitus
	Increased body weight
	Seizure
2 mechanisms	Sleep disturbance
	Ketosis
	Abnormal platelet count
	Rheumatoid arthritis
	Hematological neoplasm
1 mechanism	Abnormality of carbohydrate metabolism/homeostasis
	Abnormal glucose homeostasis
	Hypoglycemia
	Abnormal thrombosis
	Diabetic ketoacidosis
	Excessive daytime somnolence
	Reduced consciousness/confusion
	Psychosis
	Abnormality of the urinary system physiology
	Leukopenia
	Acute kidney injury
	Renal insufficiency
	Abnormality of neutrophils
	Abnormality of prenatal development or birth
	Hepatomegaly
	Skin rash
	Multiple myeloma
	Metrorrhagia
	Menstrual irregularities
	Puberty and gonadal disorders
	Abnormality of female internal genitalia
	Abnormality of the cardiovascular system
	Arteriosclerosis
	Abnormality of the systemic arterial tree
	Lymphadenopathy
	Abnormality of the lymph nodes

## Data Availability

The data used in the paper are available from the corresponding upon request due to requirements of permission and consent.

## Supplementary Materials

Supplementary Materials The top 20 overrepresented HPO terms for each drug-drug interaction mechanism is being provided in the supplementary (1).

## References

[1] Classen D. C., Pestotnik S. L., Evans R. S., Lloyd J. F., Burke J. P. (1997). Adverse drug events in hospitalized PatientsExcess length of stay, extra costs, and attributable mortality. *JAMA: The Journal of the American Medical Association*.

[2] Cullen D. J., Sweitzer B. J., Bates D. W., Burdick E., Edmondson A., Leape L. L. (1997). Preventable adverse drug events in hospitalized patients. *Critical Care Medicine*.

[3] Cullen D. J., Bates D. W., Small S. D., Cooper J. B., Nemeskal A. R., Leape L. L. (1995). The incident reporting system does not detect adverse drug events: a problem for quality improvement. *Joint Commission Journal on Quality Improvement*.

[4] Bates D. W., Spell N., Cullen D. J. (1997). The costs of adverse drug events in hospitalized patients. *JAMA: The Journal of the American Medical Association*.

[5] Bates D. W., Cullen D. J., Laird N. (1995). Incidence of adverse drug events and potential adverse drug events. *JAMA*.

[6] World Health Organization (2002). *The Importance of Pharmacovigilance*.

[7] Leaman R., Wojtulewicz L., Sullivan R., Skariah A., Yang J., Gonzalez G. Towards internet-age pharmacovigilance: extracting adverse drug reactions from user posts in health-related social networks.

[8] Noor A. (2022). Improving bioinformatics software quality through incorporation of software engineering practices. *PeerJ Computer Science*.

[9] Tatonetti N. P., Ye P. P., Daneshjou R., Altman R. B. (2012). Data-driven prediction of drug effects and interactions. *Science Translational Medicine*.

[10] Shah S. N., Gammal R. S., Amato M. G. (2021). Clinical utility of pharmacogenomic data collected by a health-system Biobank to predict and prevent adverse drug events. *Drug Safety*.

[11] Karlsson I., Zhao J., Asker L., Boström H. Predicting adverse drug events by analyzing electronic patient records.

[12] Nguyen D. A., Nguyen C. H., Mamitsuka H. (2021). A survey on adverse drug reaction studies: data, tasks and machine learning methods. *Briefings in Bioinformatics*.

[13] Lee C. Y., Chen Y.-P. P. (2021). Prediction of drug adverse events using deep learning in pharmaceutical discovery. *Briefings in Bioinformatics*.

[14] Cami A., Arnold A., Manzi S., Reis B. (2011). Predicting adverse drug events using pharmacological network models. *Science Translational Medicine*.

[15] Kovačević M., Vezmar Kovačević S., Radovanović S., Stevanović P., Miljković B. (2019). Adverse drug reactions caused by drug–drug interactions in cardiovascular disease patients: introduction of a simple prediction tool using electronic screening database items. *Current Medical Research and Opinion*.

[16] Wang G., Jung K., Winnenburg R., Shah N. H. (2015). A method for systematic discovery of adverse drug events from clinical notes. *Journal of the American Medical Informatics Association*.

[17] Chen Y.-G., Wang Y.-Y., Zhao X.-M. (2016). A survey on computational approaches to predicting adverse drug reactions. *Current Topics in Medicinal Chemistry*.

[18] Schotland P., Racz R., Jackson D. B. (2021). Target adverse event profiles for predictive safety in the postmarket setting. *Clinical Pharmacology & Therapeutics*.

[19] Chee B. W., Berlin R., Schatz B. (2011). Predicting adverse drug events from personal health messages. *AMIA Annual Symposium proceedings. AMIA Symposium*.

[20] De Rosa M., Fenza G., Gallo A., Gallo M., Loia V. (2021). Pharmacovigilance in the era of social media: discovering adverse drug events cross-relating Twitter and PubMed. *Future Generation Computer Systems*.

[21] Odom P., Bangera V., Khot T., Page D., Natarajan S. (2015). Extracting adverse drug events from text using human advice. *Artificial Intelligence in Medicine in Europe*.

[22] Pouliot Y., Chiang A. P., Butte A. J. (2011). Predicting adverse drug reactions using publicly available PubChem BioAssay data. *Clinical Pharmacology & Therapeutics*.

[23] Yamanishi Y., Pauwels E., Kotera M. (2012). Drug side-effect prediction based on the integration of chemical and biological spaces. *Journal of Chemical Information and Modeling*.

[24] Wang X., Thijssen B., Yu H. (2013). Target essentiality and centrality characterize drug side effects. *PLoS Computational Biology*.

[25] Ivanov S. M., Lagunin A. A., Poroikov V. V. (2016). In silico assessment of adverse drug reactions and associated mechanisms. *Drug Discovery Today*.

[26] Noor A., Assiri A. (2021). A novel computational drug repurposing approach for Systemic Lupus Erythematosus (SLE) treatment using Semantic Web technologies. *Saudi Journal of Biological Sciences*.

[27] Assiri A., Noor A. (2020). A computational approach to predict multi-pathway drug-drug interactions: a case study of irinotecan, a colon cancer medication. *Saudi Pharmaceutical Journal*.

[28] Köhler S., Carmody L., Vasilevsky N. (2019). Expansion of the human phenotype ontology (HPO) knowledge base and resources. *Nucleic Acids Research*.

[29] Noor A., Assiri A., Ayvaz S., Clark C., Dumontier M. (2017). Drug-drug interaction discovery and demystification using Semantic Web technologies. *Journal of the American Medical Informatics Association*.

[30] Hossain M. K., Khatun A., Rahman M., Akter M. N., Chowdhury S. A., Alam S. M. (2016). Characterization of the effect of drug-drug interaction on protein binding in concurrent administration of sulfamethoxazol and diclofenac sodium using bovine serum albumin. *Advanced Pharmaceutical Bulletin*.

[31] Lynch T., Price A. (2007). The effect of cytochrome P450 metabolism on drug response, interactions, and adverse effects. *American Family Physician*.

[32] Müller F., Fromm M. F. (2011). Transporter-mediated drug–drug interactions. *Pharmacogenomics*.

[33] Åsberg A. (2003). Interactions between cyclosporin and lipid-lowering drugs. *Drugs*.

[34] Palleria C., Di Paolo A., Giofrè C. (2013). Pharmacokinetic drug-drug interaction and their implication in clinical management. *Journal of Research in Medical Sciences : The Official Journal of Isfahan University of Medical Sciences*.

[35] Niu J., Straubinger R. M., Mager D. E. (2019). Pharmacodynamic drug-drug interactions. *Clinical Pharmacology & Therapeutics*.

[36] Dumbreck S., Flynn A., Nairn M. (2015). Drug-disease and drug-drug interactions: systematic examination of recommendations in 12 UK national clinical guidelines. *Bmj*.

[37] Bodenreider O. (2004). The unified medical language system (UMLS): integrating biomedical terminology. *Nucleic Acids Research*.

[38] Prüfer K., Muetzel B., Do H. H. (2007). FUNC: a package for detecting significant associations between gene sets and ontological annotations. *BMC Bioinformatics*.

[39] Hoehndorf R., Hancock J. M., Hardy N. W., Mallon A. M., Schofield P. N., Gkoutos G. V. (2014). Analyzing gene expression data in mice with the Neuro Behavior Ontology. *Mammalian Genome : Official Journal of the International Mammalian Genome Society*.

[40] Kaufman D. W., Kelly J. P., Johannes C. B. (1993). Acute Thrombocytopenic Purpura in Relation to the Use of Drugs. *Blood*.

[41] Curtis B. R., Divgi A., Garritty M., Aster R. H. (2004). Delayed thrombocytopenia after treatment with abciximab: a distinct clinical entity associated with the immune response to the drug. *Journal of Thrombosis and Haemostasis*.

[42] George J. N., Aster R. H. (2009). Drug-induced thrombocytopenia: pathogenesis, evaluation, and management. *Hematology*.

